# Genetically Engineered Synthetic Miniaturized Versions of *Plasmodium falciparum* UvrD Helicase Are Catalytically Active

**DOI:** 10.1371/journal.pone.0090951

**Published:** 2014-03-07

**Authors:** Abulaish Ansari, Mohammed Tarique, Renu Tuteja

**Affiliations:** Malaria Group, International Centre for Genetic Engineering and Biotechnology, Aruna Asaf Ali Marg, New Delhi, India; University of Melbourne, Australia

## Abstract

Helicases catalyze unwinding of double stranded nucleic acids in an energy-dependent manner. We have reported characterization of UvrD helicase from *Plasmodium falciparum*. We reported that the N-terminal and C-terminal fragments of PfUvrD contain characteristic ATPase and DNA helicase activities. Here we report the generation and characterization of a genetically engineered version of PfUvrD and its derivatives. This synthetic UvrD (sUD) contains all the conserved domains of PfUvrD but only the intervening linker sequences are shortened. sUD (∼45 kDa) and one of its smallest derivative sUDN1N2 (∼22 kDa) contain ATPase and DNA helicase activities. sUD and sUDN1N2 can utilize hydrolysis of all the NTPs and dNTPs, can also unwind blunt end duplex DNA substrate and unwind DNA duplex in 3 to 5 direction only. Some of the properties of sUD are similar to the PfUvrD helicase. Mutagenesis in the conserved motif Ia indicate that the mutants sUDM and sUDN1N2M lose all the enzyme activities, which further confirms that these activities are intrinsic to the synthesized proteins. These studies show that for helicase activity only the conserved domains are essentially required and intervening sequences have almost no role. These observations will aid in understanding the unwinding mechanism by a helicase.

## Introduction

Helicases catalyze the unwinding of double-stranded (ds) DNA and dsRNA or RNA secondary structure in an NTP-dependent manner. These are ubiquitous enzymes found in almost all organisms and work during a widerange of important cellular processes such as replication, recombination, repair, splicing, transcription and translation [1]–[3]. At the sequence level helicases can be classified into a number of superfamilies and they can be further classified depending on the directionality of unwinding either 5′ to 3′ or 3′ to 5′ [2]–[4]. In a recent study we have reported the genome wide analysis of helicases from the malaria parasite *Plasmodium falciparum* [5]. Earlier we have also reported that helicases could serve as potential novel drug targets for the control of malaria [6]. We have identified and characterized the parasite specific UvrD helicase from *P. falciparum* in order to develop it as a novel drug target [7], [8]. In a recent study it has been reported that the parasite specific UvrD helicase is different in a variety of Plasmodium species [9]. PfUvrD is a ∼170 kDa protein and is almost two times the size of its *Escherichia coli* counterpart [8]–[10]. Due to the large size of PfUvrD we were unable to characterize the full-length recombinant protein and we only characterized the various fragments and reported that the N-terminal and first half of the C-terminal protein contain the characteristic ssDNA-dependent ATPase and DNA helicase activities [8]. In *E. coli*, UvrD has been reported to play roles in a variety of processes such as recombination, replication, mismatch repair and nucleotide excision repair pathways [11]–[13].

Protein engineering refers to the design of de novo proteins by the substitution, addition or deletion of amino acids. This can be easily done by artificially modifying the DNA sequences which encode them so that this novel DNA can be used to produce the new proteins with desired modifications. Most common examples of protein engineering are point mutations, truncations, insertions and deletions. These modifications result into the production of inactive protein or protein with enhanced or reduced activity. The mutagenesis of the Dengue virus type 2 NS3 protein within and outside helicase motifs was done in a previous study [14]. It was observed that two mutations, both in motif I abolished both ATPase and helicase activity and two further mutations, one in motif VI and the other a clustered charged to alanine substitution abolished helicase activity only [14]. The characterization of the hepatitis E virus helicase domain showed that the helicase mutant I, with substitution in the nucleotide–binding motif I showed 30% ATPase activity and the helicase mutant II with substitutions in Mg^2+^ binding motif II showed only 50% ATPase activity. Furthermore both mutants completely lost the ability to unwind RNA duplexes [15]. In an interesting study a new bifunctional protein ‘helimerase’ was produced by engineering and physically linking *Thermoanaerobacter tengcongensis* UvrD helicase (TteUvrD) and *Bacillus stearothermophilus* DNA polymerase I large fragment (Bstpol) using a coiled-coil. It was reported that significantly longer fragments could be amplified by the helimerase in helicase-dependent amplification reactions instead of using TteUvrD and Bstpol proteins [16].

In the present study we describe engineering the UvrD helicase from *P. falciparum* and producing a modified version of it. In this synthetic UvrD (sUD) all the characteristic helicase motifs of PfUvrD are retained but the numbers of amino acids in the intervening sequence which separates these motifs are reduced. PfUvrD gene is 4326 bases which codes for a 1441 amino acids long protein, we have produced four fragments (N1, N2, C1 and C2) of this gene and ligated them and by doing this engineering we have produced a sUD protein of 389 amino acids. We have also produced the truncated versions of this protein by ligating these fragments in different combinations in order to obtain sUDN1N2, sUDN2C1, sUDC1C2, sUDN1N2C1 and sUDN2C1C2 proteins. We have biochemically characterized these proteins and report that only full-length sUD and sUDN1N2 contain the characteristic ssDNA-dependent ATPase and DNA helicase activity. This study shows that the smallest protein which demonstrates helicase activity is sUDN1N2, which is of 187 amino acids with a molecular weight of ∼22 kDa. This fragment contains the motifs Q, Ia, Ib and II of the UvrD family. The mutants of sUD and sUDN1N2 were produced by substituting two amino acids in the conserved helicase motif. Using bioinformatics and circular dichroism spectra we performed the secondary structure analysis of sUD and sUDN1N2 and the mutants’ sUDM and sUDN1N2M. We demonstrate that although there is no obvious difference in the secondary structure of mutants versus wild type proteins, the mutants’ sUDM and sUDN1N2M lose the biochemical activities such as the characteristic ATPase and thus helicase activity. These studies will advance our knowledge in understanding the unwinding mechanism by a helicase.

## Materials and Methods

### Ethics Statement

The animal studies described below were approved by the ICGEB Institutional Animal Ethics Committee (IAEC Reference No. MAL-58). ICGEB is licensed to conduct animal studies for research purposes under the registration number 18/1999/CPCSEA (dated 10/1/99).

### Cloning of Synthetic UvrD

In order to clone the sUD helicase from *P. falciparum*, the sequence was analyzed in detail. The nucleotide sequence of PfUvrD is 4326 bases and it codes for a protein of 1441 amino acids. The engineered sequence is 1170 bases and it codes for 389 amino acids long protein. The PCR amplification was done using genomic DNA as the gene is not interrupted by introns. Accordingly the following primers were synthesized to clone the N1, N2, C1 and C2 fragments. The sUD helicase gene was amplified in four fragments using the following forward and the reverse primers.

### Primers

1. UN1F: 5′-GGG*GGATCC*ATGAATGAAGATGAGGTG-3′ (BamHI)
2. UN1R: 5′-GGG*GTCGAC*ATTATTTTTATTATTAAATAATTTC-3′ (SalI)
3. UN2F: 5′-GGG*GTCGAC*TTAATTGAAACTTATCGTCTTATG-3′ (SalI)
4. UN2R: 5′-GGG*AAGCTT*CAAATTTCCTGATGTATATATTG-3′ (HindIII)
5. UC1F: 5′-GGG*AAGCTT*GAACAAACCTTTTTTAACAATAATTG-3′(HindIII)
6. UC1R: 5′-GG*GGCGGCCGC*CGTATAAAGTTGTTTTTGTATTC-3′ (NotI)
7. UC2F: 5′-GG*GGCGGCCGC*GGATTGTTTATTTTGTTTTCTTAATG-3′(NotI)
8. UC2R: 5′-GGGCTCGAGTTATATATTCATTTCATTAATAAACC-3′(XhoI)

The N1 fragment is 372 bases and codes for sUDN1 fragment from amino acid 1–124 of 14 kDa, the N2 fragment is 189 bases and codes for sUDN2 fragment of 63 amino acids (from amino acid 445–506) of 7.5 kDa, the C1 fragment is 279 bases and codes for sUDC1 fragment of 93 amino acids (from amino acid 660–752) of 11 kDa and the C2 fragment is 309 bases and codes for sUDC2 fragment of 103 amino acids (from amino acid 1339–1441) of 12 kDa respectively. The PCR conditions used were 95°C for 1 minute, 54°C for 1 min and 72°C for 2 min for the amplification of all the fragments. This was repeated for a total of 35 cycles and at the end one elongation was done at 72°C for 12 min. The PCR products were gel purified using Qiagen gel extraction kit and cloned into the pGEM-T easy vector from Promega using T-A cloning (Madison, WI, USA) and the clones were sequenced by dideoxy sequencing reactions (Macrogen, Korea). The nucleotide sequence was submitted to GenBank and the accession number for the sUDN1 fragment is JX245006, for the sUDC1fragment is JX245007 and for the sUDC2 fragment is JX245008. All these fragments were ligated to produce different combinations and the sequences were submitted to the GenBank. The accession numbers for the sUDN1N2 fragment, sUDN2C1 fragment, sUDC1C2 fragment, sUDN1N2C1 fragment, sUDN2C1C2 fragment and the complete sUD are JX245009, JX245010, JX245011, JX245012, JX245013 and JX245005 respectively.

Using the enzymes (New England Biolabs, Beverly, MA, USA) listed above all the fragments were excised from pGEMT easy clones, gel purified and subsequently cloned into pET28a+ expression vector (Novagen, Madison, WI, USA) at the appropriate sites. For protein expression, the clones were transformed into BL21 (DE3) pLysS cells. 1% of the overnight grown primary culture was inoculated in 500 ml LB (Luria Broth) and allowed to grow at 37°C. At OD 0.6 the culture was induced with 1 mM IPTG and then again allowed to grow for another 4–6 hours. The harvested cells were lysed by using lysis buffer of pH 7.8 (20 mM Tris-HCl, 250 mM NaCl, 0.1% Tween 20, 0.1% Triton 100 and the protease inhibitor cocktail from Sigma, St. Louis, MO, USA) and subsequently the cells were sonicated to lyse maximum number of cells. After centrifugation the soluble fraction was allowed to bind to pre-equilibrated Ni-NTA (Qiagen, GmbH, Germany) resin for one hour at 4°C. The column was first washed with the wash buffer (lysis buffer without detergent with 25 mM imidazole). The bound His-tagged proteins were eluted with varying (100–150 mM) concentration of imidazole in the protein buffer (20 mM Tris–HCl pH 8.0, 250 mM NaCl, 10% (v/v) glycerol and protease inhibitor cocktail from Sigma, St. Louis, MO, USA) and was checked for purity by using 10% (w/v) SDS-PAGE (sodium dodecyl sulphate polyacrylamide gel electrophoresis) electrophoresis [17].

### Site Directed Mutagenesis

The mutant of full length sUD and the fragment sUDN1N2 were generated to see the effects on their activity. Two amino acids were substituted with arginine. The conserved amino acids aspartic acid and threonine at position 62 and 63 were substituted with arginine in full length sUD and the fragment sUDN1N2. Full length sUD and the fragment sUDN1N2 were used as template to mutate these two amino acid residues in the conserved motif Ia. The sequence of the primers used is as follows and the underlined sequence denotes the mutant sequence.

### Primers

1. UMutF 5′-GCATGTCCAGGATCTGGGGCAGCATCTACATTAACAGCCAG-3′
2. UMutR 5′-CTGGCTGTTAATGTAGATGCTGCCCCAGATCCTGGACATGC-3′

The mutations were created using the standard procedures and the wild type plasmids as templates. The mutants (sUDM and sUDN1N2M) obtained were confirmed by sequencing and the sequences of the mutants were submitted to the GenBank. The accession numbers for sUDM and sUDN1N2M are KC130207 and KC130208 respectively.

### Circular Dichroism Spectra

Circular dichroism (CD) spectra were measured in order to determine the secondary structure of sUD, sUDM, sUDN1N2 and sUDN1N2M proteins. Bradford method was used to determine the protein concentration with bovine serum albumin as the standard. The final protein concentration was 0.2 mg/ml. The conditions for CD spectra recordings were 2 mm band width, 1-s averaging time, and four scans over a wavelength range of 205–250 nm at room temperature. The CD spectra were recorded on a Jasco J-715 spectropolarimeter using a 0.1-cm path-length quartz cuvette. CD spectra were also measured for all of these proteins at different pH. The protein samples were dialysed using phosphate buffer of different pH 6.5, 7.0, 7.4, 7.8, and 8.0 and CD spectra were recorded. For thermal denaturation experiment all the protein samples were gradually heated and their CD spectra were recorded at 222 nm each after 1 degree celsius interval. All thermal denaturation curves were fitted in non linear curve and the Tms were calculated.

### Generation of Polyclonal Antisera

Purified sUDN1N2 was used for the preparation of antibodies in mice using the standard protocols [17]. The polyclonal antibodies were purified as IgG fractions using protein A-Sepharose as described [17].

### Western Blot Analysis

Proteins were separated by SDS-PAGE and transferred electrophoretically to nitrocellulose membrane for western blotting as described [17]. After blocking for overnight with 3% skimmed milk in TBST (Tris buffered saline with 0.05% Tween 20), the membrane was incubated with the appropriate primary antibody (Penta-His from Qiagen, GmbH, Germany and anti sUDN1N2), for 2 h at room temperature. After washing with TBS and then TBST, the blot was incubated with the appropriate secondary antibody coupled to alkaline phosphatase (Sigma, St. Louis, MO, USA) and developed using 5-Bromo-4-Chloro-3- Indolyl Phosphate and Nitro Blue Tetrazolium purchased from Sigma.

### ATPase Assay

By using all the purified proteins such as sUDN1, sUDN2, sUDC1, sUDC2, sUDN1N2, sUDN2C1, sUDC1C2, sUDN1N2C1, sUDN2C1C2 and sUD and the mutants sUDM and sUDN1N2M the ATPase assay reaction was performed in the buffer (20 mM Tris-HCl, pH 8.0, 8 mM DTT, 1.0 mM MgCl_2_, 20 mM KCl and 16 µg/ml BSA) for 1 hour at 37°C in the presence of 10 ng of M13 mp19 ssDNA and a mixture of [γ-^32^P] ATP (Adenosine tri-phosphate) (∼17 nM) and 1 mM cold ATP [18]–[20]. The products were separated by thin layer chromatography (TLC) [18]–[20] and the plate was exposed to hyper film for autoradiography or scanned on phosphoimager. The quantitation was done using IMAGE j/geldoc software (http://rsbweb.nih.gov/ij/). For the concentration curve analysis different concentrations of sUD and sUDN1N2 proteins were used. The time course analysis was performed with a fixed concentration of sUD or sUDN1N2 and time duration ranging from 10 to 90 minutes. The quantitation was done using IMAGE j/geldoc software (http://rsbweb.nih.gov/ij/) and percentage of ATP hydrolysis was plotted as the bar diagram.

### Preparation of DNA Helicase Substrate and Helicase Assay

The helicase activity of all the purified proteins such as sUDN1, sUDN2, sUDC1, sUDC2, sUDN1N2, sUDN2C1, sUDC1C2, sUDN1N2C1, sUDN2C1C2 and sUD and the mutants sUDM and sUDN1N2M was determined by the standard strand displacement assay using the partially duplex substrate and the method described previously [8], [18], [19]. The partial duplex substrate consisted of a ^32^P-labelled 47-mer DNA oligodeoxynucleotide annealed to M13mp19 phage ssDNA. This oligodeoxynucleotide with the sequence 5′- (T)_15_GTTTTCCCAGTCACGAC(T)_15_-3′ contains 15 base-pairs of non-complementary region at both the 5′ and 3′ ends. 10 ng of the oligodeoxynucleotide was labelled at 5′-end with T4 polynucleotide kinase (PNK) (5U) (New England Biolabs) using the standard PNK buffer (New England Biolabs) and 1.85 MBq of [γ-^32^P]ATP (specific activity 222 TBq/mmol) at 37°C for one hour. This labelled oligodeoxynucleotide was then annealed using standard annealing buffer (20 mM Tris-HCl, pH 7.5, 10 mM MgCl_2_, 100 mM NaCl, 1 mM DTT) with 0.5 µg of single-stranded circular M13mp19 (+) phage DNA by heating at 95°C for 1 min, transferring immediately to 65°C for 2 min and then slow cooling to room temperature. Using gel filtration through a Sepharose 4B column (Pharmacia, Sweden) the non-hybridized oligodeoxynucleotide was removed. The reaction mixture (10 µl) containing the ^32^P-labeled helicase substrate (1000 cpm/10 µl) in appropriate buffer (20 mM Tris-HCl, pH 8.0, 8 mM DTT, 1.0 mM MgCl_2_, 20 mM KCl and 16 µg/ml BSA) and the purified protein fractions to be assayed was incubated at 37°C for 60 min. The substrate and products were separated by electrophoresis on a nondenaturing 12% PAGE, and after drying the gel was exposed to hyper film for autoradiography or scanned on phosphoimager. The quantitation of both the substrate and unwound DNA bands was done using IMAGE j/geldoc software (http://rsbweb.nih.gov/ij/) and the percent unwinding was plotted as the bar diagram.

### Preparation of Blunt End Substrate

Two kinds of blunt end substrates were made, 17 base pair blunt end substrate and normal partial duplex M13 substrate. The sequence of 17 mer oligodeoxynucleotide used for making the blunt end duplex substrate is 5′-GTTTTCCCAGTCACGAC-3′. This oligodeoxynucleotide was labelled at 5′ end and was annealed to its complementary oligodeoxynucleotide with the sequence 5′-GTCGTGACTGGGAAAAC-3′ and for another substrate it was annealed with M13 complementary region using the method described above. The substrate was purified through gel filtration and used for the assay.

### Immunodepletion Assay

IgG was purified from anti-preimmune and/or anti-sUDN1N2. For this assay aliquots of the purified sUD and sUDN1N2 were incubated with purified IgG at 0°C for 60 min. The antigen–antibody complexes were removed by the addition of protein A Sepharose beads. The supernatants were used for the ATPase and helicase activity analysis using substrate in the same way as described above.

### Determination of Km and Vmax

For this analysis helicase assay reactions for sUD and sUDN1N2 were performed using the partially duplex substrate of different concentrations (5–40 nM) in a standard reaction buffer (20 mM Tris-HCl, pH 8.0, 8 mM DTT, 1.0 mM MgCl_2_, 20 mM KCl and 16 µg/ml BSA). The amount of dsDNA and unwound ssDNA was quantified from the autoradiogram using ImageJ software (http://rsbweb.nih.gov/ij/) and used for the Km and Vmax calculations.

### Preparation of Direction Specific Substrates

The substrate consisting of long linear M13mp19 ssDNA with short duplex ends for 3′ to 5′ unwinding was prepared by first 5′-end labelling of 32-mer oligodeoxynucleotide (5′-TTCGAGCTCGGTACCCGGGGATCCTCTAGAGT-3′) and then annealing with M13mp19 ssDNA as described above. The annealed substrate was digested with SmaI and purified by gel filtration through 1 ml of Sepharose 4B. For preparing a 5′ to 3′ direction-specific substrate, the 32-mer oligodeoxynucleotide was first annealed to M13mp19 ssDNA using annealing buffer (20 mM Tris-HCl, pH 7.5, 10 mM MgCl_2_, 100 mM NaCl, 1 mM DTT) and then labelled at 3′-OH end in appropriate buffer with 50 µCurie [α-^32^P]dCTP and 5 units of DNA polymerase I (large fragment) at 23°C for 20 min. The incubation was continued for an additional 20 min at 23°C after increasing the dCTP to 50 mM using unlabelled dCTP. This resulting duplex substrate was digested with SmaI and purified by gel filtration through 1 ml Sepharose 4B.

## Results and Discussion

### Sequence Analysis of sUvrD

UvrD belongs to superfamily 1 of helicases. In a recent study we have reported the detailed characterization of UvrD homologue from the malaria parasite *P. falciparum* [8]. PfUvrD is about two times the size of *E. coli* UvrD and as reported earlier it contains long insertions in between the conserved domains [8]. In the present study we report the characterization of a synthetic UvrD helicase which was made based on the sequence of the full length PfUvrD. The alignment of the sUD with the PfUvrD is shown (Figure S1). This alignment was done using Clustal Omega (http://www.ebi.ac.uk/Tools/msa/clustalo/). The results show that all the conserved motifs are present and the intervening linker sequences between the various motifs are considerably truncated. The 1A, 1B, 2A and the 2B domains are also depicted in the figure (Figure S1, red, blue, green and yellow boxes, respectively). An alignment of the complete amino-acid sequence of *E. coli* UvrD and sUD using Clustal Omega (http://www.ebi.ac.uk/Tools/msa/clustalo/) is shown (Figure S2). The engineered sUD protein is about half the size of *E. coli* UvrD and the 1A, 1B, 2A and the 2B domains are also depicted in the figure (Figure S2, red, blue, green and yellow boxes, respectively). We used the strategy shown in Figure 1 for the synthesis of the sUD (Figure 1A). The sequence and positions of various motifs in PfUvrD is shown in Figure 1B. The complete gene for *sUD* was amplified in four fragments and then these fragments were ligated to obtain the full-length gene. The sUDN1 fragment contains motifs Q, Ia, Ib and first 25 amino acids of the intervening sequence between motifs Ib and II (Figure 1C). The sUDN2 fragment contains motif II and the last 25 amino acids of the intervening sequence between motifs Ib and II and the first 25 amino acids of the intervening sequence between motifs II and III (Figure 1C). The sUDC1 fragment contains the last 25 amino acids of the intervening sequence between motifs II and III, motifs III and IV and the first 25 amino acids of the intervening sequence between motifs IV and V (Figure 1C). The sUDC2 fragment contains the last 25 amino acids of the intervening sequence between motifs IV and V, motifs V and VI till the end (Figure 1C). All of these fragments were amplified and used separately for the analysis and also these fragments were ligated to produce the complete sUD of 389 amino acids (Figure 1D).

**Figure 1:** Sequence and domain organization of UvrD. A. The detailed domain organization of *P. falciparum* UvrD helicase. The conserved sequences of each domain are written inside the boxes. The text in blue refers to the names of various conserved domains and the numbers refer to the amino acids separating the various domains and the length of N- and C-terminal extensions. This figure is not drawn to scale. B. The strategy used for constructing the various fragments. The numbers in red refer to the reduced number of amino acids in between the domains. The details of all the fragments are listed. C. Domain organization of full length sUD. D. Complete amino acid sequence of synthetic UvrD (sUD). The sequence of conserved domains is written in bold letters. See also Figures S1 and S2.

### Molecular Modelling of sUD Structure

For structural modelling the sequence of the engineered sUD was submitted to the Swissmodel homology-modelling server (http://swissmodel.expasy.org/). A total of six models were obtained and four models covered the smaller areas of sUD ranging from 69 to 148 amino acids only but only one model covered a larger range (amino acid 32–388) of the sUD sequence. Therefore this model which was built using E. coli helicase as template was analyzed in detail. The residues 32 to 388 of the engineered sUD sequence showed ∼15% sequence identity to this E. coli helicase [10]. The structural modelling of the sUD was therefore done using the known crystal structure of this homologue as the template (PDB number 2is6-A at http://www.rcsb.org/pdb/explore). The ribbon diagram of the template is shown in Figure 2A and the predicted structure of sUD is shown in Figure 2B. When the modelled structure of sUD and the template were superimposed, it is clear that these structures superimpose partially (Figure 2C). Similarly for structural modelling the sequence of sUDN1N2 was submitted to the Swissmodel homology-modelling server (http://swissmodel.expasy.org/). Two models were obtained and these models covered the areas of sUDN1N2 ranging from 71 to 125 amino acids. Model 1 which was built using PcrA DNA helicase from B. stearothermophilus as template was analyzed in detail [21]. sUDN1N2 primary sequence residues 32 to 121 showed ∼28% sequence identity to the PcrA DNA helicase from B. stearothermophilus [21]. The structural modelling of the sUDN1N2 was therefore done using the known crystal structure of this homologue as the template (PDB number 3pjr-A at http://www.rcsb.org/pdb/explore). The ribbon diagram of the template is shown in Figure 2E and the predicted structure of sUDN1N2 is shown in Figure 2F. When the modelled structure of sUDN1N2 and the template were superimposed, it is clear that these structures superimpose partially (Figure 2G). These results suggest that the removal of intervening sequences has no effect on the overall structure of the protein. Molecular graphic images were produced using the UCSF Chimera package (http://www.cgl.ucsf.edu/chimera) from the Resource for Biocomputing, Visualization, and Informatics at the University of California, San Francisco (supported by NIH P41 RR-01081) [22]. The PDB files of modelled sUD and sUDN1N2 proteins were subjected to PDBsum server (http://www.ebi.ac.uk/thornton-srv/databases/pdbsum/Generate.html) for further secondary structure analysis [23]. It is noteworthy that α-helix, β-sheets, β-turns, and coils are present in both sUD and sUDN1N2 proteins (Figure 2D and 2H, respectively). The overall predicted secondary structure of sUD protein shows the presence of 19 α-helices, 24 β-turns, 20 helix-helix interactions, 4 γ-turns, and 9 strands (Figure 2D). On the other hand the overall predicted secondary structure of sUDN1N2 protein shows the presence of only 4 α-helices, 4 β-turns, 3 helix-helix interactions and 4 γ-turns (Figure 2H).

**Figure 2:** Structure modelling of synthetic UvrD. A–C. sUD sequence was submitted to Swissmodel server and the structure was obtained. A. Template B. sUD C. superimposed image. D. Secondary structure of sUD. E–G. sUDN1N2 sequence was submitted to Swissmodel server and the structure was obtained. E. Template; F. sUDN1N2; G. superimposed image. D. Secondary structure of sUDN1N2.

The nucleotide sequence of *sUD* gene is 1170 bases and it codes for a protein of 389 amino acids with a calculated molecular weight of 45 kDa. For the amplification of full-length sUD fragments genomic DNA from *P. falciparum* 3D7 strain was used with the primer pairs UN1F and UN1R, UN2F and UN2R, UC1F and UC1R, and UC2F and UC2R to amplify the sUDN1, sUDN2, sUDC1 and sUDC2 fragments respectively. Each of these fragments were amplified and cloned as described in materials and methods section. Besides these, various combinations of these fragments such as sUDN1N2, sUDN2C1, sUDC1C2, sUDN1N2C1, sUDN2C1C2 were ligated and used for analysis. Finally all the four fragments such as sUDN1, sUDN2, sUDC1 and sUDC2 were ligated to obtain the full-length sUD (Figure 1C and D).

### Protein Purification of All the Fragments

The expression clones analogous to each fragment such as fragment sUDN1, sUDN2, sUDC1, sUDC2, sUDN1N2, sUDN2C1, sUDC1C2, sUDN1N2C1, sUDN2C1C2 and sUD were transformed into *E. coli* BL21 (DE3) pLysS strain and the recombinant proteins were purified using method described in materials and methods section. The SDS–PAGE analysis of the purified proteins showed that all the proteins are almost pure and homogeneous preparations (Figure 3A, lane 1 and 2 contain purified sUD and sUDN1N2, respectively, lanes 5–8 contain sUDN2C1, sUDC1C2, sUDN2C1C2 and sUDN1N2C1, respectively and Figure 3B, lanes 1–4 contain sUDN1, sUDN2, sUDC1, and sUDC2, respectively). The purified fractions were further checked by western blot analysis using anti-his antibodies and only a single band in each of the purified fraction was detected (Figure 3C, lane 1 and 2 contain purified sUD and sUDN1N2, respectively, lanes 5–8 contain purified sUDN2C1, sUDC1C2, sUDN2C1C2, and sUDN1N2C1, respectively and Figure 3D, lanes 1–4 contain purified UDN1, sUDN2, sUDC1, and sUDC2, respectively). These purified recombinant proteins were used for all of the assays described in the subsequent sections. The purified sUDN1N2 protein was also used for the production of polyclonal antibodies in mice.

**Figure 3:** SDS PAGE and Western blot analysis. A and B. Coomasie blue stained gel. Lane M in A and B are protein molecular weight markers and the proteins loaded in each lane are written on top of the gels. C and D. Western blot analysis. Lane M in C and D are protein molecular weight markers and the proteins loaded in each lane are written on top of the gel.

### Determination of Secondary Structure of Proteins

The PSIPRED protein structure prediction server was used to determine the secondary structure of all the four proteins sUD, sUDM, sUDN1N2 and sUDN1N2M [24], [25]. The amino acid sequence of all the four proteins was submitted to the server at http://bioinf.cs.ucl.ac.uk/psipred and the results were downloaded. The results clearly show that all of these proteins mainly consist of helical structure (Figure 4A–D). Furthermore there is no obvious structure difference between sUD and sUDM (Figure 4A and B) and between sUDN1N2 and sUDN1N2M (Figure 4C and D), respectively.

**Figure 4:** A–D. Secondary structure representation. The protein sequences of sUD, sUDM, sUDN1N2 and sUDN1N2M were submitted to the server at http://bioinf.cs.ucl.ac.uk/psipred/and the secondary structures were determined. The graphs in A–D represent the structures of sUD, sUDM, sUDN1N2 and sUDN1N2M, respectively. E. Circular dichroism (CD) spectra of sUD, sUDM, sUDN1N2 and sUDN1N2M. F-G. CD spectra of sUD and sUDM, and sUDN1N2 and sUDN1N2M, respectively at different temperature.

For determining the secondary structure of proteins CD spectra is an excellent method [26]. The α-helix, β-sheet, and random coil structures each have a characteristic shape and magnitude of CD spectrum. The approximate fraction of each secondary structure type that is present in any protein can thus be determined by analysing its far-UV CD spectrum [26]. After modification or mutation in protein, CD spectrum is also used for comparison of conformations between native and mutant forms. Therefore CD spectra of all the four proteins such as sUD, sUDM, sUDN1N2 and sUDN1N2M were measured in order to determine their secondary structures using the method described in materials and methods section. The results clearly show that there is no random coil in all of these proteins. The peaks in negative range (troughs) at 208 to 222 nm in the CD spectra suggest that all of these proteins have α-helix-rich secondary structure (Figure 4E). The data clearly indicate that both the full length proteins sUD and sUDM are rich in α-helix as compared to their truncated counterparts sUDN1N2 and sUDN1N2M (Figure 4E). The data further indicate that little shift in band is observed between the spectra of sUD versus its mutant sUDM but there is no significant difference between the spectra of sUDN1N2 versus its mutant sUDN1N2M. These data suggest that mutations have no detectable effect on the conformation of the protein.

The CD spectra of all the four proteins were also measured at pH 6.5, 7.0, 7.4, 7.8 and 8.0. The data indicate that on increasing pH of the buffer all four proteins are stabilized (Figure S3). This may be explained as at lower pH, more hydrogen ions affect charges of amino acid and unfold proteins. It is well known that CD spectra can be used to determine whether the melting temperature (Tm) or slope of a transition changes when mutations are present. Tm is a parameter to measure stability of proteins [27]. In order to determine the effects of mutations on protein stability, the CD spectra of all the four proteins were measured as a function of temperature. The data clearly indicate that there is no significant difference in the curves of sUD versus sUDM (Figure 4F) and sUDN1N2 versus its mutant sUDN1N2M (Figure 4G). Tm of sUD, sUDM, sUDN1N2 and sUDN1N2M are 68.16, 65.2, 53.1, and 52.2°C, respectively. These observations suggest that in the present study the two amino acid mutations have no significant measurable effect on the stability of proteins. Furthermore it is interesting to note that the Tm of sUD and sUDN1N2 are reasonably different (68.16 versus 53.1).

### Characterization of ATPase and DNA Helicase Activities

The ssDNA-dependent ATPase activity of all the purified protein fragments was tested using standard assay conditions as described in materials and methods section in the presence of traces of radiolabelled ATP, 1 mM cold ATP and purified proteins. The results indicated that except the purified sUDN1N2 and sUD none of the other fragments such as sUDN1, sUDN2, sUDC1, sUDC2, sUDN2C1, sUDC1C2, sUDN1N2C1, and sUDN2C1C2 showed any ATPase activity (Figure 5A, lanes 2–16 and Figure 5B, lanes 2–7, respectively). The concentration-dependence of ATPase activity was tested by using 5 nM to 100 nM of sUD and 50 to 1000 nM of sUDN1N2 proteins. The percent release of radioactive inorganic phosphate (Pi) from [γ^32^P] ATP was measured. The results clearly showed that sUD (Figure 5C, lanes 1–8) and sUDN1N2 (Figure 5E, lanes 1–7) contain concentration dependent ATPase activity. The ATPase reaction using 80 nM of purified sUD and 600 nM of purified sUDN1N2 at different time interval was done in order to study the time dependence of ATPase activity. The percent release of radioactive Pi from [γ^ 32^P] ATP showed linearity up to 100 minutes in both sUD and sUDN1N2 (Figure 5D and 5F, lanes 1–8, respectively). The standard helicase strand-displacement assay measures the unwinding of ^32^P-labelled DNA fragment from a partially duplex nucleic acid. Since there was no ATPase activity in any of the other proteins, therefore the DNA unwinding activity of only sUDN1N2 and sUD was determined using the standard strand-displacement assay. The DNA unwinding activity using different concentration of purified sUD (5 to 100 nM) and sUDN1N2 (50 to 1000 nM) and optimal assay conditions as described in materials and methods section with 1000 cpm of the substrate in buffer having 1 mM ATP, 1 mM MgCl_2_ and 75 mM KCl was tested. It is interesting to note that sUD showed the concentration-dependent and time-dependent helicase activity (Figure 6A and 6B, lanes 1–8 and lanes 1–7, respectively). Similarly sUDN1N2 also showed the concentration-dependent and time-dependent helicase activity (Figure 6C and 6D, lanes 1–8 and lanes 1–8, respectively). It is interesting to note that the ATPase and helicase activities of sUD are about 10 fold more as compared to sUDN1N2. About 10 times more concentration of sUDN1N2 as compared to sUD is required to obtain same enzymatic activities (Figure 5C and 5E and 6A and 6C). One of the possible reasons for this may be the structural difference between these two synthetic proteins. In the previous section we have reported that the Tm of sUD and sUDN1N2 are different and this might be one of the reasons that more concentration of sUDN1N2 is required to obtain same enzymatic activity.

**Figure 5:** Analysis of ATPase activity. A. Lane 1, sUD, lanes 2–4, increasing concentration of sUDN1, lanes 5–7, increasing concentration of sUDN2, lanes 8–10, increasing concentration of sUDC1, lanes 11–13, increasing concentration of sUDC2, and lanes 14–16, increasing concentration of sUDN2C1. B. Lane 1 contains sUD, lanes 2–3, increasing concentration of sUDC1C2, lanes 4–5, increasing concentration of sUDN1N2C1, lanes 6–7, increasing concentration of sUDN1N2C2. C. Concentration dependent ATPase activity of sUD, Lanes 1–8 are increasing concentration of sUD and concentration are labelled at top of the autoradiogram. D. Time dependence of ATPase activity of sUD. The time of incubation in minutes is mentioned at the top of the autoradiogram and C is the control reaction without enzyme. E. Concentration dependent ATPase activity of sUDN1N2, Lanes 1–7 are increasing concentration of sUDN1N2 and concentration are labelled at top of the autoradiogram. F. Time dependence of ATPase activity of sUDN1N2. The time of incubation in minutes is mentioned at the top of the autoradiogram. C in panels A–F is the control reaction without enzyme. see also Figure S4.

**Figure 6:** Analysis of helicase activity. A. Helicase activity of sUD. The quantitative enzyme activity data from the autoradiogram are shown and the concentration of sUD is also written on the X axis of the bar diagram. B. Time-dependence of helicase activity of sUD. The quantitative enzyme activity data from the autoradiogram are shown and the time is written on X-axis. C. Helicase activity of sUDN1N2. The quantitative enzyme activity data from the autoradiogram in C are shown and the concentration of sUDN1N2 is written on the X axis of the bar diagram. D. Time-dependence of helicase activity of sUDN1N2. The quantitative enzyme activity data from the autoradiogram are shown and the time is written on X-axis. In panels A–D, lane C is reaction without enzyme and lane B is heat denatured substrate. see also Figure S3 and S4.

Since only the sUD and sUDN1N2 showed helicase activity therefore it was interesting to find if physical mixture of these individual protein fragments will show any unwinding activity. Therefore the helicase activity of the physical mixture of sUDN1 and sUDN2 and all the four fragments such as sUDN1, sUDN2, sUDC1 and sUDC2 was tested. The results were interesting since none of the combination showed any unwinding activity (Figure S4). These results suggest that all the helicase domains should be on a single polypeptide for the enzyme to be active.

### Immunodepletion of ATPase and Helicase Activities

Purified sUD and sUDN1N2 were allowed to react separately with IgGs purified from the pre-immune sera and from the sera of the mice immunized with sUDN1N2 using the method described in materials and methods section. The immunodepleted supernatants were checked for ATPase and helicase activities. The results showed that the ATPase activity of sUD (Figure 7A, lanes 1–3) and sUDN1N2 (Figure 7B, lanes 1–3) was depleted with the specific anti-sUDN1N2 antibodies. On the contrary the samples treated with pre-immune IgG for both sUD and sUDN1N2 showed concentration-dependent ATPase activity (Figure 7A, lanes 4–8 and Figure 7B, lanes 4–8, respectively). Similar results were obtained with helicase activity also. The results showed that the helicase activity of sUD (Figure 7C, lanes 5–8, respectively) and sUDN1N2 (Figure 7D, lanes 5–8, respectively) using helicase substrate was also depleted with the specific sUDN1N2 antibody. But the samples treated with pre-immune IgG for both sUD and sUDN1N2 showed concentration-dependent helicase activity (Figure 7C, lanes 1–4 and Figure 7D, lanes 1–4, respectively). These data further confirm that the ATPase and helicase activities are due to the purified sUD and sUDN1N2 proteins and not due to any contamination in the purified preparations.

**Figure 7:** Analysis of ATPase and helicase activities after immunodepletion. A. ATPase activity of sUD. Lanes 1–3, reactions with increasing concentration of sUD pretreated with immune IgG, lanes 4–8 reactions with increasing concentration of sUD pretreated with pre-immune IgG. B. ATPase activity of sUDN1N2. Lanes 1–3, reactions with increasing concentration of sUDN1N2 pretreated with immune IgG, lanes 4–8 reactions with increasing concentration of sUDN1N2 pretreated with pre-immune IgG. Lane C in A and B is reaction without protein. C. Helicase activity of sUD. Lanes 1–4, reactions with increasing concentration of sUD pretreated with pre-immune IgG, lanes 5–8, reactions with increasing concentration of sUD pretreated with immune IgG. D. Helicase activity of sUDN1N2. Lanes 1–4, reactions with increasing concentration of sUDN1N2 pretreated with pre-immune IgG, lanes 5–8 reactions with increasing concentration of sUDN1N2 pretreated with immune IgG. In panel C and D, lane C is reaction without protein and lane B is heat treated substrate. In each panel the quantitative data from the autoradiogram are also shown.

### ATPase and Helicase Activities of Mutants

The mutants, sUDM and sUDN1N2M, which contained mutation in the conserved motif Ia were generated as described in materials and methods section. The purity of these mutants was checked using SDS-PAGE and western blot analysis along with the wild type sUD and sUDN1N2 (Figure 3A, lanes 3 and 4 contain sUDM and sUDN1N2M, respectively and Figure 3C, lanes 3 and 4 contain sUDM and sUDN1N2M, respectively). In the previous sections we have reported that the biophysical properties of the mutants are almost similar to their wild type counterparts (Figure 4A–G). In order to check the effect of mutations on the enzymatic activities, the ATPase and helicase activities of these mutants’ sUDM and sUDN1N2M were checked. None of the mutants, sUDM or sUDN1N2M, showed any ATPase activity (Figure S5A, lanes 2–7 and Figure S5B, lanes 2–8, respectively) or helicase activity (Figure S5C, lanes 1–2 and lanes 5–6, respectively). These results further indicate that although the mutations in the helicase conserved domain have no measurable effect on the biophysical properties but the mutations abolish the ATPase and helicase activity of sUDM and sUDN1N2M, therefore the activities observed in the wild type forms, sUD and sUDN1N2 are authentic.

### Determination of Km and Vmax for the Helicase Activity

Helicase assay reactions were performed using different concentrations of DNA duplex substrate (5–40 nM) in a standard reaction buffer keeping constant concentration of sUD (40 nM) and sUDN1N2 (800 nM). The amount of dsDNA and unwound ssDNA was quantified as described in materials and methods section. A conventional hyperbolic dependence of the rate of reaction on substrate concentration was obtained, such that the rate of substrate unwinding was initially linear and later saturated with increasing substrate concentrations that gave best-fit to the Michaelis–Menten equation. The Km and Vmax of helicase activity for sUD and sUDN1N2 was measured by using Sigma plot software (http://www.sigmaplot.com/). Nonlinear regression analysis of this data yielded a Km value of 1.195 nM and 2.096 nM for sUD (Figure 8A) and sUDN1N2 (Figure 8B), respectively. The Vmax value is 1.421 nM/min/ng and 1.274nM/min/ng for sUD and sUDN1N2, respectively. The Km values are comparable to the values reported earlier for PfUDN and PfUDC1 [8] but Vmax values are higher as compared to values reported earlier for PfUDN and PfUDC1 [8].

**Figure 8:** Kinetics of helicase activity. A. sUD and B. sUDN1N2. Helicase assay reactions were performed using different concentrations of substrate and keeping constant concentration of sUD and sUDN1N2. Km and Vmax values were calculated from the plot.

### Advanced Characterization of Unwinding Activity

Further characterization of unwinding activity was done using sUD and sUDN1N2. It is well known that specific nucleotides are required for helicase for its unwinding activity. Therefore to check if there is any specific nucleotide requirement for unwinding activity by sUD and sUDN1N2, their helicase activity was measured with different deoxynucleotide triphosphates and nucleotide triphosphates. It is interesting to note that sUD and sUDN1N2 showed the unwinding activity with all the dNTPs and NTPs such as dCTP, CTP, dGTP, GTP, dATP, ATP, dTTP and UTP used for the reaction (Figure 9A, lanes 1–8 and 9B, lanes 1–8, respectively). But sUD and sUDN1N2 did not show any unwinding activity in the absence of any NTP or dNTP (Figure 9A, lane C and 9B lane C, respectively). Further evaluation was done to determine the optimum concentration of ATP for the unwinding activity of sUD and sUDN1N2. The results showed that unwinding activity of sUD and sUDN1N2 was maximal at 1.5 mM ATP concentration and it did not increase further on increasing the ATP concentration to 5.0 mM (Figure 9C and 9D, lanes 1–7, respectively) but in the absence of ATP, sUD and sUDN1N2 did not show any unwinding activity (Figure 9C and 9D, lane C respectively). These data are also similar to the results obtained with PfUDN, which showed activity in all the deoxynucleotide triphosphates and nucleotide triphosphates but its activity was maximal at 2.5 mM ATP concentration [8].

**Figure 9:** Determination of nucleotide-dependence of helicase activity. A–B. Nucleotide requirement of helicase activity of sUD (A) and sUDN1N2 (B). Helicase activity of sUD and sUDN1N2 in the presence of NTP/dNTPs written on top of the gel. Lane C is enzyme reaction in the absence of any NTP or dNTP and B is heat denatured substrates. C–D. Helicase activity of sUD (C) and sUDN1N2 (D) using varying concentration of ATP written on top of the gel. Lane C is enzyme reaction without any ATP and B is heat denatured substrate. In panel A–D, the quantitative enzyme activity data from the autoradiogram are shown.

In order to further explore the substrate specificity of sUD and sUDN1N2 a 17 base pair blunt end duplex substrate and an M13 partial duplex substrate, without overhangs were also tested for the DNA unwinding activity. Blunt end duplex substrate had blunt ends but contained matching core sequence and same duplex length as normal substrate (17 basepair) so that any differences in competence of unwinding due to sequence differences could be nullified. The M13 partial duplex substrate had 17 base pair complementary oligonucleotide sequence annealed to M13 ssDNA. The assay was done using the method described in the previous section. The results clearly show that sUD and sUDN1N2 unwind the M13 17 base pair duplex substrate in concentration dependent manner (Figure 10A, lanes 1–6, and 10B, lanes 1–6, respectively). It was interesting to note further that sUD and sUDN1N2 unwind the blunt end duplex DNA substrate also in concentration dependent manner (Figure 10C, lanes 1–6, and 10D, lanes 1–6, respectively). These data are similar to the results obtained with PfUDN, which showed activity with blunt end substrate also [8].

**Figure 10:** Unwinding activity analysis of sUD and sUDN1N2 with different substrates. The structure of the substrate used is shown. Asterisk (*) denotes the ^32^P-labeled end. A. Lanes 1–6 are the reactions with increasing concentration of sUD. B. Lanes 1–6 are the reactions with increasing concentration of sUDN1N2. C. Lanes 1–6 are the reactions with increasing concentration of sUD. D. Lanes 1–6 are the reactions with increasing concentration of sUDN1N2. In panel A–D, lane C is reaction without enzyme and lane B is heat treated substrate.

### Determination of Direction of Unwinding by sUD and sUDN1N2

Helicases are known to preferentially unwind nucleic acids in a polar fashion by moving unidirectionally on the bound strand in a duplex. The strand to which the enzyme binds and moves defines the direction of unwinding by a helicase. The unwinding activity of both sUD and sUDN1N2 was tested by using two different direction-specific substrates, one specific for the 5′ to 3′ and the other for the 3′ to 5′ direction, prepared as described in materials and methods section. By using both the direction-specific substrates the DNA unwinding activity of different concentrations of sUD and sUDN1N2 proteins was determined. The results clearly show that both sUDN1N2 and sUD (Figure 11A, lanes 1–4 and lanes 5–8, respectively) were unable to show the activity with the 5′ to 3′ direction-specific substrate. On the other hand it is obvious from the results that sUDN1N2 and sUD (Figure 11B, lanes 1–4 and lanes 5–8, respectively) were able to unwind the 3′ to 5′ direction-specific duplex substrate in an efficient manner indicating that both of these contain unidirectional DNA unwinding activity. The helicase activity with the direction specific substrate was also directly proportional to the concentration of sUD and sUDN1N2 used in the reaction (Figure 11B, lanes 1–4 and lanes 5–8 respectively). As reported earlier PfUDN also contains unidirectional 3′ to 5′ direction activity [8].

**Figure 11:** Representation of direction specific unwinding activity. A. 5′ to 3′ direction specific substrate. Lanes 1–4, increasing concentration of sUD, lanes 5–8, increasing concentration of sUDN1N2. B. 3′ to 5′ direction specific substrate. Lanes 1–4 contain increasing concentration of sUD, lanes 5–8, increasing concentration of sUDN1N2. In panel A and B, the structure of the substrate is shown and asterisk (*) denotes the ^32^P-labeled end and lane C is reaction without protein and lane B is heat denatured substrate. Quantitative data of figure B are shown and the concentration used is written on X axis of bar diagram.

Overall in the present study we have reported the construction and characterization of a synthetic helicase and its smaller derivative, which contain the characteristic ATPase and DNA helicase activities. To the best of our knowledge this is a novel study and reports the characterization of the smallest helicase.

## Supporting Information

Figure S1 **Comparison of amino acid sequence of** ***P. falciparum*** **PfUvrD and sUD.**
(TIF)

Figure S2 **Comparison of amino acid sequence of** ***Escherichia coli*** **EcUvrD and sUD.**
(TIF)

Figure S3 **CD spectra of sUD, sUDN1N2, sUDM and sUDN1N2M at different pH.**
(TIF)

Figure S4 **Helicase activity analysis of purified sUD proteins.**
(TIF)

Figure S5 **Helicase and ATPase activities of synthetic mutant proteins.**
(TIF)
